The article "Clinical Observation of Botulinum Toxin Injection in the Treatment of Focal Dystonia and Muscle Spasm" was retracted in 2023. Reasons: unreliable results or conclusions; lack of ethics approval or compliance; concerns about the data; concerns about the peer review.

# Clinical Observation of Botulinum Toxin Injection in the Treatment of Focal Dystonia and Muscle Spasm

**DOI:** 10.1155/2022/1495807

**Published:** 2022-09-05

**Authors:** Zhen Zhang

**Affiliations:** Neurology, Panjin Central Hospital, Panjin, 124013 Liaoning, China

## Abstract

Dystonia and muscle spasms are a group of common and unfavorable clinical neurological symptoms. The use of botulinum toxin (BTX-A) abroad has achieved good results in the treatment of various movement disorders characterized by involuntary or abnormal muscle contractions. It is expected to open up a new field for the treatment of myelodysplastic syndromes (MDs) such as focal dystonia and muscle spasm. There are theoretical and practical implications for the diagnosis and development of some effective neurological treatments. The efficacy of BTX-A in the treatment of various focal dystonia and muscle spasm disorders is as follows: symptoms were improved to varying degrees after injection of Botox or botulinum toxin type A (CBTX-A), but Botox or CBTx. There was no significant difference in the efficacy of A. 30.4% of patients had complete remission, 57.8% had significant remission, and 8.9% had partial remission. Among them, HFS and BS had the best curative effect, and the symptoms were significantly improved by 95.3% and 89.4%, respectively. The efficacy of CD was also satisfactory, with 75.5% of the patients showing significant improvement in symptoms, followed by Meg/OMD (OMD) with 73.3% and SD with 3.3%. The efficacy of WC is poor, and functional improvement is uncertain. Other forms of focal dystonia and spasticity also showed significant functional improvement in 60% of patients. Most patients start to see effects within 1 week after BTX-A injection, symptoms gradually improve, and the bridge of curative effect is reached in 2-4 weeks, and the healing effect lasts for about 3-5 months on average. The overall severity of adverse effects was not severe and resolved spontaneously within a few days to ten weeks, with the most concerning complications being ptosis and dysphagia.

## 1. Introduction

Dystonia and muscle spasms are a group of common and unfavorable clinical neurological symptoms. The patient's symptoms are obvious, often aggravated by activities, causing severe pain and suffering to the patient's body and mind. Dystonia is a functional disease second only to Parkinson's in incidence. The most common clinical disorder is focal dystonia, such as blepharospasm, spastic torticollis, writing spasm, and spastic anxiety disorder. Most symptoms are initially hidden and may gradually get worse. Due to the complex etiology, changeable symptoms, few clear and durable curative effects of previous treatments, difficulty in quantifying functional impairment, and difficulty in examination and evaluation, it has been underemphasized for a long time. Clinical studies of CBTX-A for the treatment of eyelid and hemifacial spasm have been reported, but there is no attempt to treat spasmodic torticollis, Meige, writing spasm, and comparison with foreign preparations. To enable the research carried out in this work, botulinum toxin was piloted to treat various neuropathic MDs characterized by involuntary or abnormal muscle contractions. The study was greatly encouraged by comparing the results of botulinum toxin in the treatment of spasticity. It is hoped to open up a new field for the treatment of MDs such as regional dystonia and muscle spasm. It has important theoretical and practical significance for evaluating and developing some effective treatment methods. The purpose of this study was to explore the methods, doses, clinical indications, complications, and long-term efficacy of botulinum toxin treatment. It also conducts a comparative analysis of Chinese and American preparations, further studies electrophysiological changes, deepens understanding, and promotes the application of botulinum toxin in the treatment of neurological diseases.

Botulinum neurotoxins are a class of potent protein neurotoxins produced by the anaerobic bacterium botulinum and are the most toxic toxins known to date. In recent years, botulinum toxin has sometimes caused many civilian poisoning incidents and can also be abused in military warfare as a terrorist and biological agent. Therefore, the study of botulinum toxin has attracted the attention of researchers all over the world. There is currently no effective treatment for botulism, and horse serum extracts are mainly used for treatment. However, horse serum has disadvantages such as the risk of viral contamination and allergic reactions. In recent years, with advances in genetic engineering in the production of engineered humanized antibodies, the use of a single antibody has been found to be ineffective. Combinations of multiple monoclonal antibodies may have positive neutralizing and protective effects. The article examines the combination of monoclonal antibodies against different botulinum toxin epitopes, and the screening of the study is the combination of antigenic epitope analysis and antibody screening. Antibody screening is guided by antibody analysis, and the identification of corresponding antigenic epitopes and receptor-binding monoclonal antibody epitopes in antibody screening lays the foundation for the development of antibody therapy and antibody detoxification mechanisms.

In the past ten years, botulinum toxin has taken the place of traditional medicine. Botulinum toxin has been used to treat a variety of movement disorders. And it is considered to be the most effective drug for focal dystonia, especially the first-line treatment of spastic torticollis. The short-term effectiveness of botulinum toxin in the treatment of spastic torticollis has been confirmed, generally taking effect within 7-10 days. However, spasticity is a chronic disease process, and most patients require a long-term treatment. Therefore, it has certain clinical practical value to explore the long-term efficacy of botulinum toxin treatment, its influencing factors, and safety.

## 2. Related Work

In the clinical research of focal dystonia and muscle spasm, there are also many research results of world experts. Saito et al. made splints for patients that allow stretching and improve finger muscle tone and contractures. After the patient received 5 doses of botulinum toxin type A, the proximal muscle spasm of the upper extremity gradually decreased [1]. Kaymak et al. believed that intramuscular botulinum toxin (BoTX) is the first-line treatment for cervical dystonia. However, after BoTX application, poor treatment results and some side effects have been reported [2]. Douglas et al. believed that ADCY5 mutations should be considered in the presence of overt myoclonic dystonia and that ADCY5-related dyskinesia may manifest differently in a family [3]. Asahi et al. believed that abdominal thalamotomy is effective in patients with focal task-specific dystonia, but only in patients with upper extremity symptoms [4]. However, the limitations of the above studies are large, and the clinical effects of botulinum toxin injections on focal dystonia and muscle spasm were tested.

Fischoff and Silvia reported changes in pain intensity in patients 19 years of age and older in a randomized controlled trial (RCT) comparing botulinum toxin type A (BoNT-A) with placebo for trigeminal neuralgia (TN) [5]. Marcelissen et al. consulted many reports of clinical experience with BoNT-A, especially in patients with neurogenic detrusor hyperactivity. It was recently approved for idiopathic overactive bladder [6]. Campanati et al. found that botulinum toxin has also been experimentally used in many other skin diseases recently and achieved good results [7]. However, the above research was not used because the data was not public and the credibility was not high.

## 3. Structure and Function of BoNT/A

Botulinum neurotoxins are a class of potent protein toxoids produced by anaerobic Clostridium botulinum. According to their different antigenicity, they can be divided into various subtypes. A toxin molecule can inactivate a neuron, and its LD50 ranges from 0.1 to 1 ng/kg body weight, resulting in a very low dose of poisoning in humans. Only 0.1-1 *μ*g can cause muscle relaxation paralysis of the whole body and eventually lead to respiratory failure and death [8]. The subtypes of botulinum toxin molecules share many structural similarities (Figure 1). In the early stage of molecular formation, it is a single-chain polypeptide with a size of about 150 kDa, which has zinc endopeptidase activity and acts on nerve cells. It consists of three functional regions: catalysis, transport, and binding. The three are linearly arranged, and the three functional domains are independent; the catalytic region is a light chain with a molecular weight of 50 kDa, a compact spherical structure composed of *α*-helix and *β*-sheet; the transport domain is the amino terminus of the heavy chain with a molecular weight of 50 kDa. It is mainly composed of *α*-helix; the binding region is the carboxyl terminus of the heavy chain with a molecular weight of 50 kDa, which is composed of two subunits, and the carboxyl terminus binds to the target cell. Both the heavy and light chains are linked by a disulfide bond [9].

The poisoning mechanism of BoNT/A is shown in Figure 2 [10]. When botulinum toxin molecules are secreted, they form polymers with their auxiliary proteins. In the gastric acid environment, the auxiliary proteins can prevent the botulinum toxin molecules from being enzymatically hydrolyzed. When the botulinum toxin molecules enter the intestinal lumen, the weak alkaline environment makes the accessory proteins separate from the botulinum toxin molecules. The botulinum toxin molecules pass through the small intestine epidermis and enter the blood circulation and lymphatic circulation system. It acts on the neuromuscular junction and prevents the release of acetylcholine, causing muscle relaxation paralysis [11]. The process of botulinum toxin molecules from intestinal epithelial cells to cholinergic nerves can be divided into four steps. The first step is the recognition and binding of target cells, during which experts put forward the dual receptor theory. The second step is internalization. The botulinum toxin molecule enters the cell through endocytosis under the action of BoNT/AHn, and the acidic environment exposes the hydrophobic fragment of the botulinum toxin molecule to the molecular conformation surface. It enables the toxin to be embedded within the lipid bilayer; the fourth step is to block the release of neurotransmitters. BoNT/AL acts on the substrate SNARE protein to prevent the release of acetylcholine, causing muscle relaxation paralysis [12].

### 3.1. Synaptic Vesicle Proteins

Synaptic vesicle 2 is a transmembrane glycoprotein that is widely expressed in endocytic and synaptic vesicles. SV2 contains a hydrophobic transmembrane moiety, which controls the release of neurotransmitter biomass through intracellular vesicle endocytosis, maintains synaptic vesicle homeostasis, and participates in the regulation of synaptic connection muscles [13]. Studies have shown that SV2, SV2A, SV2B, and SV2C can utilize these three isoforms as the BoNT/A receptor of TM48LR and the pocket synapse between TMR7 and TMR7. After that, the structure of the BoNT/A-SV2C complex was analyzed by means of crystal analysis, and the amino acid residues S1142, M1144, T1145, T1146, and Y1149 were finally determined to have direct interaction between BoNT/A and SV2C, as shown in Figure 3. The structural analysis of the BoNT/A-SV2C complex more objectively confirmed the conclusion that SV2C is a BoNT/A receptor [14]. Although the number of SV2C on the surface of nerve cells is small, it has a high affinity for toxins. In the mechanism of botulism, it is responsible for binding to toxins and mediating toxin internalization [15].

### 3.2. Fibroblast Growth Factor Receptor 3

Fibroblast growth factor receptor 3 is a tyrosine kinase receptor and a member of the fibroblast growth factor receptor family. There were a total of 806 amino acids having relative molecular weight of 110 kD~135 kD [16]. It is mainly distributed in fibrous and connective tissues and is involved in life activities such as signal transduction, tissue repair, and cell regeneration, differentiation, and apoptosis [17]. As shown in Figure 4, FGFR3 consists of three parts: extracellular domain, transmembrane domain, and intracellular domain. The extracellular domain is the ligand binding domain and the transmembrane domain is the protected hydrophobic domain; the intracellular domain can also be divided into a cytoplasmic very variable access membrane domain and two active tyrosine kinase domains [18]. By analyzing the crystal structure of BONT/A, it is found that it has homology with the structure of fibroblast growth factor, so it is speculated that the receptor of FGFs can also become the receptor of BONT/A. Further experiments demonstrated that the ligand BONT/A could act as an agonist for the receptor FGFR3 to phosphorylate it. The ligands FGF1, FGF2, and FGF9 compete with BONT/A for binding to the receptor FGFR3. It blocks the uptake of toxins by cells, and it is concluded that FGFR3 plays a key role in the process of cell-specific uptake of BONT/A. The mutation scheme formulated according to the mutation principle is shown in Table 1 [19].

According to the experimental results, the screened small peptides Nos. 20, 21, and 37 were further truncated to shorten the binding range of the receptor on BoNT/AHC [20]. Truncations of small peptides are designed on the basis that a minimum of 7 amino acids is required to form the binding site. The binding of small peptides 20 and 21 to receptor FGFR3 was relatively high. Based on this, it is speculated that the overlapping region of these two small peptides is more likely to be the receptor binding site. Therefore, the sequence of the truncated peptide 20-21 was designed as NSGWKVSLNY. No. 37 has the strongest binding force among the 46 peptides, so three truncated peptides were designed based on the middle 5 amino acids of No. 37: 37-1MFKLDGC, 37-2KLDGCRD, and 37-3MFKLDGCRD. The detection of the binding ability of the truncated peptide to the receptor was evaluated by indirect ELISA. The synthesized 20-21, 37-1, 37-2, and 37-3 small peptides were dissolved in PBS and then diluted to 10 *μ*g/ml with coating buffer. 10 *μ*g/ml BoNT/AHC was added to the positive wells, and coating buffer was added to the blank wells, and the protein FGFR3D23 was diluted with PBST to a concentration of 10 *μ*g/ml. The wells showed a positive reaction compared with the positive wells and the negative wells. The experimental results were analyzed with the P/Y value greater than 2.1 as the criterion for positive reaction. Its findings still meet this requirement, as shown in Figure 5. That is to verify that the ligand BoNT/A can interact specifically with the receptor FGFR3 [21].

### 3.3. Preparation of BoNT/AHC Complex Crystals with FGFR3

Domain 2/3 of the protein FGFR3 is the binding domain of BoNT/A, so we expressed the protein FGFR3D23 and identified FGFR3D23 as inclusion body expression, and the inclusion body needs to be renatured into a soluble protein. The renaturation of inclusion bodies is a uniform protein with a similar natural conformation, which is conducive to the formation of complex crystals. As shown in Figure 6, the renatured FGFR3D23 protein conformation is uniform. However, no crystals were detected in the late protein BoNT/AHC and FGFR3D23, so subsequent experiments could not be performed.

In this paper, the successfully sequenced plasmids were transformed into BL21(DE3), coated on LB(Amp) plates, and single colonies were picked and cultured at 37°C 220 rpm to midlogarithmic phase. After low temperature induction by adding IPTG, the expression of protein BoNT/AHCC was identified by 12.5% polyacrylamide gel electrophoresis. Electrophoresis results showed that the target protein was expressed in the form of inclusion bodies. The target protein was dissolved in a solution containing 8 M urea and then subjected to Ni-IDA affinity purification. After SDS-PAGE detection, samples with higher purity were collected for renaturation. In this paper, renaturation was carried out by dialysis, and the purified samples were placed in imidazole gradient dilution renaturation solution and dialyzed each concentration for 6 hours. Finally, it was dialyzed into 2 M urea renaturing solution and then transferred to storage solution. The binding ability of truncated mutants BoNT/AHC, BoNT/AHCN, and BoNT/AHCC to receptor FGFR3 at different concentrations was detected by indirect ELISA. In this paper, grouped *t* test was performed on the results, and the results showed that there was no difference in the binding of BoNT/AHC and BoNT/AHCN to receptors (*p* = 0.064 > 0.05), the binding of BoNT/AHC and BoNT/AHCC to the receptor was different (*p* = 0.006 < 0.05), and the binding of BoNT/AHCN and BoNT/AHCC to the receptor was different (*p* = 0.022 < 0.05).  Figure 7 shows the binding curves of the three truncation mutants to the receptor FGFR3 at different concentrations. From this result, it was concluded that the HCN region on the ligand BoNT/A was responsible for binding to the receptor FGFR3.

Six cases were not treated according to the prescribed rehabilitation program, 4 cases of recurrence without follow-up, 2 cases of respiratory and obstructive pulmonary disease, and 2 cases of recurrence after 6 months, and the last 78 cases were included in the study. The most common recurrence group was group A, with a total of 21 cases, and the BONT-A injection group was groups B, C, and D, with 19 cases, 18 cases, and 20 cases, respectively. The limbs correspond to 37, 35, 34, and 35, respectively. There was no significant difference in the incidence of spastic cerebral palsy and GMFCS among the four groups (*p* > 0.05), and there was no significant difference in the distribution of MAS among the four groups before treatment, leprosy (*F* = 0.35, *p* = 0.91 > 0.05). Compared with the initial treatment, the MAS scores of each group were significantly decreased at any time after treatment (*F* = 14.16, *p* < 0.05). The MAS score after each treatment was lower than that of group A (*p* < 0.05), and the decrease was most obvious at 1 month. Then, it increased slightly with the prolongation of treatment time and was higher than the level before treatment 12 months after treatment (*F* = 0.22, *p* < 0.05). The comparison of group B, group C, and group D showed that postoperative MAS grades were not always significantly different (*F* = 14.17, *p* > 0.05). Tables 2 and 3 show the comparison of MAS scores in the four groups before and after treatment.

There was no significant difference in iEMG values between the four groups in the passive state of sEMG before treatment (*F* = 0.62, *p* = 0.75 > 0.05). The IEMG values in the passive state of sEMG decreased significantly at each time point after treatment (*F* = 99.70, *p* < 0.05). And it may be stable at 6 months and 12 months after treatment (*F* = 16.4, *p* > 0.05). The comparison shows that there is no significant difference in iEMG value in each passive state of sEMG after treatment (*F* = 7.52, *p* > 0.05).

### 3.4. Molecular Docking in the Epitope-Restricted State of Receptor FGFR3

Based on the results of the preliminary docking analysis in this paper, for the binding mode of cluster 5 and cluster 7, the nonpeptide 20, 21, and 27 regions of FGFR3 were set to block state. And it was molecularly docked with BoNT-AHc in the block state; for the binding mode of cluster 4, the D2 domain of FGFR3 was set to the block state.

(1) $$\begin{array}{c} \text{ZDOCL Score}>15,\text{ZRANK Score}<-30,\text{Intermolecular Bumps},\\ \text{SI}=\frac{\text{test grou}{\text{p}}_{\text{OD}}‐\text{blank backgroun}{\text{d}}_{\text{OD}}}{\text{unstimulated grou}{\text{p}}_{\text{OD}}‐\text{blank backgroun}{\text{d}}_{\text{OD}}}. \end{array}$$

In order to ensure that each step in the construction process is accurate, it is necessary to carry out the corresponding enzyme digestion identification of the intermediate vector in the construction process. It will also be verified by sequencing to further confirm the constructed plasmid.

(2) $$\begin{array}{c} \text{pABE}293-\text{scDEC},\text{carrier},\\ \text{pABE}293-\text{scDEV},\text{vector digestion}\left(\text{BamH}/\text{Xho}4.4\text{kb}+830\text{bp}\right),\\ \text{pTIG}-\text{scDEC},\text{carrier}. \end{array}$$

Firstly, the scDEC gene was excised from the pGH-Yu-scDEC vector and connected to the pABE293 vector to construct pABE293-scDEC. The restriction enzyme digestion identification was correct.

(3) $$\begin{array}{c} \text{pTIG}-\text{scDEC vector digestion}\left(\text{BamH I}/\text{Xho I}5.6\text{kb}+830\text{bp}\right),\\ \text{pTIG}-\text{scDEC}-\text{AHc},\text{carrier},\\ \text{pTIG}-\text{scDEC}-\text{AHc},\text{vector digestion}\left(\text{BamHI}/\text{XhoI}5.6kb+2.1\text{kb}\right). \end{array}$$

In the last step, the fusion gene scDEC-AHc was excised from the pTIG-scDEC-AHc vector and connected to the pVAX1 vector. The restriction digestion identification was correct, and the plasmid construction was completed.

(4) $$\begin{array}{c} \text{pVAX}1-\text{scDEC}-\text{AHc},\text{carrier},\\ \text{pVAX}1-\text{scDEC}-\text{AHc},\text{vector digestion}\left(\text{BamHI}/\text{XhoI}2.9\text{kb}+2.1\text{kb}\right). \end{array}$$

## 4. Botulinum Toxin for Focal Dystonia and Muscle Spasms

The experimental samples were selected from nearly 1,000 patients who voluntarily received injections of botulinum toxin or CBTX-A in a hospital neurology clinic. A total of 785 patients had at least one follow-up visit after treatment. It includes physical therapy, acupuncture, integrated traditional Chinese and Western medicine, and surgical treatment, all of which are ineffective or recur. The general condition of the patients at the time of initial diagnosis is shown in Table 4. Among them, 488 cases of hemifacial spasm, 106 cases of different degrees of facial paralysis, 85 cases of blepharospasm, 26 cases of Meg's syndrome, 4 cases of dystonia, and 159 cases of spastic torticollis. Sixty-four patients (40.3%) had cervical pain, 42 (26.4%) had primary or postural tremor, and 10 had segmental or generalized dystonia. Nine cases had a history of taking antipsychotic drugs before the onset, 2 cases had a family history of torticollis, and 3 cases had spastic dysarthria, all of which were adduction type. One case had systemic dystonia. Five cases had writing spasm, and 1 case had familial hereditary Parkinson's disease; occupations are doctor, secretary, preauditor, office cadre, and accountant, all related to excessive writing. There were 7 cases of other forms of focal dystonia, including 1 case of bilateral upper extremity dystonia caused by Wilson's disease, 4 cases of unexplained unilateral dystonia, and 1 case of exercise-induced diaphragmatic muscle spasm and 1 case of abdominal muscle spasm. There were 5 cases of spasticity caused by stroke, myelopathy, and cerebral palsy, 1 case of pain spasm caused by multiple sclerosis, and 2 cases of local disease-induced muscle tension.

Patients usually follow specific guidelines to find the best results, accepting a sitting, neutral, and stable posture. It uses 1 ml or 5 ml disposable syringes to sterilize alcohol for cell injection, dose adjustment, size, volume, and flexibility manipulation depending on muscle spasm. It is injected using a coated Tenol needle, a double-needle EMG needle, or manual therapy. It is suitable for patients with spastic muscle problems that are difficult to diagnose with actual surgery, or patients with poor initial response. Elevating muscle status is performed during electromyography (EMG) testing, where the orbicularis oculi muscle can be applied to the affected area along with the skin via cell injection. Orbicularis oris injection requires more caution to reduce side effects such as ulceration and avoid midline injections to prevent ptosis. The total dose is 12.5-10 U. In the case of spastic torticollis, the most commonly injected muscles are the head and neck muscles, sternocleidomastoid, trapezius, scapula, and skeletal muscles (Figure 8). Multiple injections were used in the muscle, the dose of each cell injection should not exceed 100 U, and the total amount of each injection should not exceed 400 U. Each treatment consists of 1-2 injections. Usually the first treatment requires more time and effort to achieve the best results. For CD patients with mixed type and poor response to initial treatment, the application of EMG in the treatment process is very helpful. The same is true for patients who are obese, have a history of surgery, or require injections into the deep neck muscles.

For the observed cases, the most common preinjection treatment was acupuncture combined with traditional Chinese medicine, benzodiazepines, and antiepileptic drugs. The exploratory oral drug treatments described in this article all have mild or transient side effects. Increasing the dose can improve local symptoms; however, there are systemic side effects that patients cannot tolerate, and surgical treatment has a specific effect, but the trauma is obvious, there is a specific risk, and there is a considerable probability of recurrence. One patient with torticollis underwent accessory nerve clamping, amputation of quadratus muscle, and partial amputation of sternocleidomastoid muscle 3 times. The patient relapsed after less than 2 months of symptom remission, and Table 5 shows the treatment the patient used before the BTx-A injection.

The grading changes of BS patients after Botox and CBTX-A injections are shown in Figure 9. After Ridit analysis, *p* < 0.01, the differences were extremely significant. Blepharospasm is reduced or disappeared after treatment, and wrinkles around the eyes are reduced. Some patients' visual function improved significantly, and their self-care ability improved. Symptoms improved significantly in the botulinum toxin group and CBTX-A group by 86.7% and 90.9%, respectively. Patient-reported subject improvement averaged 7.7 and 7.6 points, respectively. The adverse reactions after HFS and BS injections are shown in Table 6. Generally speaking, these adverse reactions are not serious, such as incomplete closure of palpebral fissures, expressionless face, tight closure of both sides, and difficulty in closing eyes, and eye irritation symptoms refer to local pain, tearing, dryness, and discomfort at the injection site. There were 2 cases of digestive tract reaction and 2 cases of skin rash in the CBTX-A group. The above symptoms do not require special treatment, they will improve on their own within 1-18 weeks, and most patients can accept it. The most concerning complication is ptosis. The incidence rates of Botox and CBTX-A groups were 5.4-7.1% (8/147 cases in Botox group and 30/422 cases in CBTX-A group) and returned to normal within 2-14 weeks. The analysis of factors related to ptosis after BTx-A injection showed that only the age of the patients and the medication dose had statistical significance in those with ptosis and those without ptosis. Eyelid ptosis is generally older, and the injection dose is relatively large.

The most common postinjection complications in CD patients are local pain, neck muscle weakness, and dysphagia. The pain from the injection will disappear within a few days, and neck muscle weakness is most common in patients with injections into the head and neck muscles of the spine and the deep extensor muscles of the neck. Difficulty swallowing with head up, drinking is usually caused by discomfort or numbness in swallowing. These adverse reactions developed rapidly within 1 to 12 weeks. In the CBTx-A group, there were 3 cases of rash within a few days after the injection, which disappeared within two weeks after the treatment with the allergy drug. One patient, 54 years old, male, and CD patient, developed nausea and vomiting on the day of injection of CBTX-A300U. If the patient is fatigued and has difficulty breathing, the patient should be observed in the emergency department, infused for 5 days, and improved after a few weeks of rest. No serious complications occurred, and the specific data are shown in Figure 10.

The treatment of dystonia has always been a difficult problem for neurologists. Symptoms of localized muscle spasms can be aggravated by mental factors and thus have a functional color, which can easily be mistaken for the performance of sores. But experience has shown that these patients are rarely cured by psychotherapy. The etiology of most dystonias is unknown, and there is currently no effective drug or radical surgical method. Therefore, it is important for doctors and patients to screen for low-risk first-line treatments. Because BTX-A is used to treat many diseases or symptoms characterized by involuntary, abnormal, or excessive muscle contraction, it has become a preventive treatment method for various diseases due to its strong curative effect, reliable curative effect, and low side effects. It is the method of choice for dystonia due to its simplicity, such as spastic torticollis, blepharospasm, Meige syndrome, occupational spasm, spastic dysarthria, and hemifacial spasm. It also has numerous reports of BTX-A in the treatment of spasticity, tremor, twitching, muscle formation, muscle motility, painful myotonia, and unexplained muscle hypertrophy.

## 5. Discussion

Muscle tone and muscle spasms are permanent motion sickness syndromes caused by impaired brain development. During leg cramps, muscle stiffness, increased muscle tone, and hyperreflexia may occur. And with the degree of pain, they cannot balance during exercise, and their posture is different from normal people. In difficult situations, they cannot move or even take care of themselves. It can have a severe impact on daily life, cause severe psychological burden, and make it harder for family members to care for it. Clinical rehabilitation should focus on addressing motor developmental disorders and postural deficits. The main goal of treating lower extremity muscles in SP patients is to maintain a relatively stable hand posture to prevent secondary soft tissue contractions. At present, due to the lack of specific methods for the treatment of spasm, BONT-A injection has the advantages of rapid antispasmodic effect, strong selectivity, and few side effects. It is widely used clinically.

Common methods of BoNT-A guidance include freehand stretching, EMG localization, electrical stimulation localization, MRI localization, CT localization, and ultrasound guidance. Reverse posture is comfortable, easy, and painless, but not effective in targeting deep, thin muscles. EMG injection method has its own specific injury, but the family may not accept it, but it can be seen in the muscle position. The correct positioning can be connected through the neuromuscular connection, but the correspondence between the position and the injection point is not high. Electroinjection method easily identifies the muscle movement points and easily stimulates the patient. However, the cost is high and the operation is incompatible, such as exposure to ionizing radiation during CT diagnosis and limited diagnostic area. It results in limited BoNT-A injection guidance. Ultrasound has been used in the field of human vision since it was first used to scan brain structures. It clearly identifies the muscles, glands, and blood vessels of the nerves, and the location is very precise, preventing improper injections.

According to the severity of spasticity, assessment results, and clinical manifestations, different doses of BoNT-A were selected for injection. The recommended dose of botulinum toxin for the treatment of spasticity in humans is between 0.5 and 6 U/kg. The American Society of Reconstructive Medicine's botulinum toxin guidelines for the treatment of limb spasticity in adults recommend that an adult dose of 600 U be injected at one time, and each injection site should not exceed 50 U. In addition, the recommended doses for pediatric injections are pediatric GMFCSI~IV16-20 U/kg and pediatric GMFCSV12-16 U/kg. A comparative study of 120 patients with spastic paralysis showed that compared with the lower dose, the younger the age, the better the effect and the higher the dose (2 U/kg, 3 U/kg), the more obvious the effect. 90 children with spastic cerebral palsy were selected for clinical observation. After injection, GMFM and MAS were used for evaluation, and the clinical efficacy of 1, 2, and 3 months was monitored. The results showed no difference in recovery rates and overall development of spasticity, reducing the financial burden. However, the article does not discuss muscle and muscle morphology and the effectiveness of seasonal injections. Although high doses of BoNT-A have been reported to disrupt muscle microarchitecture in animal experiments, the effects of high-dose injections on pediatric muscles cannot be ruled out. And because the maximum dose of adult lower extremity muscle is 6 U/kg, based on safety considerations, this study selected a higher dose of BoNT-A 5 U/kg per injection. Considering the economy, drug resistance, and potential adverse reactions, this study selected 3-5 U/kg for injection, and 3-5 injection points were selected for each target muscle to facilitate the enhanced diffusion of the drug.

## 6. Conclusion

BoNT-A injections combined with restorative therapy can reduce spasticity and increase physical strength over conventional therapy alone; BoNT-A injections can be varied between doses of 3 U/kg, 4 U/kg, and 5 U/kg depending on appropriate preset settings. Specifically, there was no difference between relief of spasticity and improvement in physical function, changes in spastic muscles, and improvement in all physical functions. BoNT-A injection is safe and effective without side effects. In conclusion, BTX-A injection is the best drug group for the treatment of myocardial infarction and local dystonia without destroying muscle growth. It included drug therapy muscle changes and side effects of different BoNT drugs, which were better than the normal recovery group with no significant difference. However, this study still has limitations, such as enrollment age, number of patients, and duration. Botulinum toxin is also an effective method for the treatment of muscle spasm in patients. Local injection of BTX is used to treat local dystonia, hemifacial spasm, abductor muscle, and other nervous system pain symptoms. They provide safe, easy, effective, and reliable treatment to eliminate symptoms and eliminate physical and mental problems in patients. Botulinum toxin can improve patients' lives as one of the first effective and stand-alone therapies, and there is no doubt that it has effective therapeutic applications. At the same time, we also need to recognize the various flaws and problems that need to be addressed.

## Figures and Tables

**Figure 1:** Schematic diagram of the molecular structure of BoNT.

**Figure 2:** Mechanism of botulinum toxin poisoning—schematic diagram of blocking neurotransmitter release.

**Figure 3:** Structure of SV2C and BoNT/A binding site.

**Figure 4:** Structure of fibroblast growth factor receptor 3.

**Figure 5:** Interaction of BoNT/AHC and FGFR3.

**Figure 6:** FGFR3D23 renaturation identification.

**Figure 7:** Analysis of the binding ability of the three BoNT/A mutants to the receptor FGFR3 at different concentrations.

**Figure 8:** Distribution of affected premuscles in CD patients.

**Figure 9:** Changes in Cohen's grading of BS after BTX-A injection.

**Figure 10:** Adverse reactions of Botox and CBTx-A injections in the treatment of CD.

**Table 1:** Mutation scheme.

Mutant	Mutation site	Original amino acid	Mutated amino acid
AHT1	1296-1248	RNND	YATAA
AHT2	1265-1254	RVY	AGCAAA
AHT3	1232-1254	QEI	AAATA
AHT4	1117-1220	KQR	GAAAA
AHT5	1254-4582	MI	AAA
AHT6	1127-1165	NR	AAAA
AHT7	1165-1184	NNS	ATA
AHT8	1127-1165	SNLGN	YAA
AHT9	921-923	VKNK	AAATA
AHT10	1035-1048	IKQR	GAAAA
AHT11	1245-1554	LNNE	AAA
AHT12	1296-1542	QEI	AAAA
AHT13	1174-1184	KQR	ATA
AHT14	1265-1297	MI	YAA
AHT15	1296-1263	FHQ	AAA
AHT16	1236-1254	FNN	AAA
AHT17	1296-1248	WYN	AASA
AHT18	1265-1254	RQIE	TMAAA
AHT19	1232-1254	RSSRT	SAT
AHT20	885-887	SNH	AAATA
AHT21	917-921	FNSIS	GAAAA
AHT22	1054-1065	LNNE	AAA
AHT23	1064-1066	QEI	AAAA
AHT24	1117-1220	KQR	ATA
AHT25	1254-4582	MI	YAA
AHT26	1127-1165	NR	AAPA
AHT27	921-923	NNS	YATAA
AHT28	1035-1048	SNLGN	AGCAAA
AHT29	1146-1147	VKNK	AAATA
AHT30	993-936	IKQR	GAAAA

**Table 2:** Balance test of clinical data of four groups of treatment plans for children with hamstring spasm.

Factor	Group A	Group B	Group C	Group D	*p* value
Spastic hemiplegia	7	3	5	3	0.45
Spastic diplegia	12	11	8	12	
Spastic quadriplegia	6	5	2	7	
GMFCS classification					
Class I	5	5	5	4	0.476
Class II	8	4	7	6	
Class III	7	8	8	7	

**Table 3:** Comparison of MAS grades before and after treatment in four groups of children.

Group	Number of limbs	Before therapy	After treatment			
			January	March	June	December
Group A	26	2.0 ± 0.5	3.8 ± 0.6	2.7 ± 0.3	2.7 ± 0.6	2.7 ± 0.6
Group B	24	2.9 ± 0.6	3.4 ± 0.7	1.6 ± 0.5	1.2 ± 0.5	1.5 ± 0.4
Group C	24	2.0 ± 0.3	3.5 ± 0.6	1.8 ± 0.7	1.3 ± 0.4	2.6 ± 0.4
Group D	25	2.0 ± 0.4	3.5 ± 0.6	2.7 ± 0.3	1.4 ± 0.8	2.6 ± 0.2

**Table 4:** General information of the patient.

Diagnosis	Number of cases	Male: Female	Age	Disease duration
			X ± SD‚ range	X ± SD‚ range
HFS	488	198 : 290	48.3 ± 12.6, 12~17	62.2 ± 62.8, 1~480
BS	85	39 : 65	53.2 ± 12.1, 45~82	3.2 ± 59.5, 2~324
Meige/OMD	30	52 : 12	55.1 ± 12.2, 21~73	46.0 ± 52.4, 4~240
CD	158	21 : 45	45.5 ± 14.6, 5~73	43.3 ± 58.3, 1~360
SD	3	76 : 74	23.3 ± 17.9, 32~55	64.0 ± 52.3, 36~156
WC	5	3 : 5	61.8 ± 14.5, 41~69	42.6 ± 96.5, 15~240
Other focal	7	4 : 4	25.3 ± 23.7, 12~62	35.4 ± 23.9, 5~60
Spasticity, etc.	9	4 : 3	21.4 ± 12.5, 12~58	67.8 ± 73.9, 12~240
Total	785	347 : 428	32.7 ± 13.2, 5~82	51.7 ± 60.9, 1~480

**Table 5:** Treatments used by patients before BTx-A injection.

	Antiepileptic drugs	Baclofen	Traditional Chinese medicine	Facial nerve block	Operation
HFS	151		347	125	21
BS	14	3	18		4
Meige	15	6	22		4
CD	26	7	122		17
SD		5	3		
WC			2		
Other Dyst	6		1		
Spasticity		3	5		
Total	212	24	520	125	47

**Table 6:** Adverse reactions after BTX-A injection in HFS and BS.

	CBTX-A	Botox	*p* value
Incomplete closure of palpebral fissures	23 (12.6)	92 (26.3)	>0.05
Facial muscle weakness or worsening of the original facial paralysis	36 (24.6)	80 (21.6)	>0.05
Eye irritation symptoms	23 (15.6)	50 (12.6)	>0.05
Drooping eyelids	18 (4.6)	31 (5.6)	>0.05
General malaise, flu-like symptoms	7 (5.6)	17 (4.5)	>0.05
Blurred vision	2 (2.6)	18 (3.5)	>0.05
Gastrointestinal reaction	3	5 (2.6)	
Rash	2	4 (2.1)	

## Data Availability

No data were used to support this study.

## References

[1] Saito K., Saito Y., Hirota K., Matui H., Hase K. (2021). Long-term effects of combined botulinum toxin treatment and rehabilitation on upper limb muscle spasms: a case report. *Journal of Physical Therapy Science*.

[2] Kaymak B., Kara M., Güray E. (2018). Sonographic guide for botulinum toxin injections of the neck muscles in cervical dystonia. *Physical Medicine and Rehabilitation Clinics of North America*.

[3] Douglas A. G. L., Andreoletti G., Talbot K. (2017). ADCY5-related dyskinesia presenting as familial myoclonus-dystonia. *Neurogenetics*.

[4] Asahi T., Taira T., Ikeda K., Yamamoto J., Sato S. (2018). Full recovery from drummer's dystonia with foot and arm symptoms after stereotactic ventro-oral thalamotomy: a case report. *Acta Neurochirurgica*.

[5] Fischoff D. K., Silvia S. (2018). Botulinum toxin for facial neuralgia. *Evidence-Based Dentistry*.

[6] Marcelissen T. A. T., Rahnama’i M. S., Snijkers A., Schurch B., De Vries P. (2017). Long-term follow-up of intravesical botulinum toxin-A injections in women with idiopathic overactive bladder symptoms. *World Journal of Urology*.

[7] Campanati A., Martina E., Giuliodori K., Consales V., Bobyr I., Offidani A. (2017). Botulinum toxin off-label use in dermatology: a review. *Skin Appendage Disorders*.

[8] Vergara-Fernández O., Salgado-Nesme N., Navarro-Navarro A., Rangel-Ríos H. A. (2017). Meta-analysis of botulinum toxin injection for chronic anal fissure: healing rates controversies. *Techniques in Coloproctology*.

[9] Baum R. P., Langbein T., Singh A. (2018). Injection of botulinum toxin for preventing salivary gland toxicity after PSMA radioligand therapy: an empirical proof of a promising concept. *Nuclear Medicine & Molecular Imaging*.

[10] Awan K. H. (2017). The therapeutic usage of botulinum toxin (Botox) in non-cosmetic head and neck conditions - an evidence based review. *Saudi Pharmaceutical Journal*.

[11] Buonocore M., Demartini L., Mandrini S., Dall'Angelo A., Dalla Toffola E. (2017). Effect of botulinum toxin on disabling neuropathic pain: a case presentation suggesting a new therapeutic strategy. *PM & R : The Journal of Injury, Function, and Rehabilitation*.

[12] Esch B., Wegner I., Stegeman I. (2017). Effect of botulinum toxin and surgery among spasmodic dysphonia patients. *Otolaryngology and Head and Neck Surgery*.

[13] Santoro A., Fontana A., Miscio A. M., Zarrelli M. M., Copetti M., Leone M. A. (2017). Quarterly repeat cycles of onabotulinumtoxinA in chronic migraine patients: the benefits of the prolonged treatment on the continuous responders and quality-of-life conversion rate in a real-life setting. *Neurological Sciences*.

[14] Collins L., Sathiananthamoorthy S., Fader M., Malone-Lee J. (2017). Intermittent catheterisation after botulinum toxin injections: the time to reassess our practice. *International Urogynecology Journal*.

[15] Licia G., Eleonora G., Emanuela S. (2018). Onabotulinumtoxin A for chronic migraine with medication overuse: clinical results and changes in catastrophising attitude. Preliminary data. *Neurological Sciences*.

[16] Kim B. W., Kim H. J., Hyun J. K., Kim S. Y., Kim T. U. (2018). Botulinum toxin injection in the treatment of postextubation dysphagia: a case report. *Annals of Rehabilitation Medicine*.

[17] Warner T., Dystonia T. (2017). Dystonia. *British Medical Bulletin*.

[18] Foley J. A., Vinke R. S., Limousin P., Cipolotti L. (2017). Relationship of cognitive function to motor symptoms and mood disorders in patients with isolated dystonia. *Cognitive and Behavioral Neurology*.

[19] Almeida L., Martinez-Ramirez D., Ahmed B. (2017). A pilot trial of square biphasic pulse deep brain stimulation for dystonia: the BIP dystonia study. *Movement Disorders Official Journal of the Movement Disorder Society*.

[20] Raoofi S., Khorshidi H., Najafi M. (2017). Etiology, diagnosis and management of oromandibular dystonia: an update for stomatologists. *Journal of Dentistry*.

[21] Ma J., Wang L., Yang Y. M., Mao C. H., Wan X. H. (2018). Novel SERAC1 mutations in a Chinese patient presenting with parkinsonism and dystonia. *Neurological Sciences*.

